The article "MNAT1 is overexpressed in colorectal cancer and mediates p53 ubiquitin-degradation to promote colorectal cancer malignance" was retracted in 2021. Reasons: duplicated images; unreliable data; lack of ethics approval or compliance; concerns about the data.

# MNAT1 is overexpressed in colorectal cancer and mediates p53 ubiquitin-degradation to promote colorectal cancer malignance

**DOI:** 10.1186/s13046-018-0956-3

**Published:** 2018-11-26

**Authors:** Shan Zhou, Jinping Lu, Yuejin Li, Chan Chen, Yongqiang Cai, Gongjun Tan, Zhengke Peng, Zhenlin Zhang, Zigang Dong, Tiebang Kang, Faqing Tang

**Affiliations:** 1 Department of Clinical Laboratory, Hunan Cancer Hospital &The affiliated Cancer Hospital of Xiangya School of Medicine, Central South University, Changsha, 410013 China; 2 Department of Clinical Laboratory, Zhuhai Hospital, Jinan University, Zhuhai, 519000 Guangdong China; 3 Hormel Institute, University of Minnesota, 801 16th Avenue NE, Austin, MN 55912 USA; 4 State Key Laboratory of Oncology in South China and Department of Experimental Research, Sun Yat-sen University Cancer Center, Guangzhou, 510060 Guangdong China

**Keywords:** MNAT1, Colorectal cancer, p53, Ubiquitin, Tumorigenesis

## Abstract

**Background:**

MNAT1 (menage a trois 1, MAT1), a cyclin-dependent kinase-activating kinase (CAK) complex, high expresses in various cancers and is involved in cancer pathogenesis. However, mechanisms underlying its regulation in carcinogenesis are unclear.

**Methods:**

The tissue microarray of colorectal cancer (CRC) was used to evaluate MNAT1 expressions in CRC tissues using immunohistochemistry, CRC cell lines were also detected MNAT1 expression using Western-blotting. MNAT1 and shMNAT1 vectors were constructed, and transfected into CRC cells. Cell growths of the transfected cells were observed using MTT and colony formation. The affects of MNAT1 on p53 expression were analyzed using Western-blotting and Real-time PCR. Immunoprecipitation assay was used to analyze the interaction p53 and MNAT1, and Western-blotting was used to test the effects of MNAT1 on p53 downstream molecules. The apoptosis of CRC cells with MNAT1 or shMNAT1 were analyzed using flow cytometry. BABL/c athymic nude mice were used to observe the effect of MNAT1 on CRC cell growth in vivo*.*

**Results:**

MNAT1 was found to be overexpressed in CRC tissues and cells, and MNAT1 expressions in CRC tissue samples were associated with CRC carcinogenesis and poor patient outcomes. *MNAT1*-knockin increased CRC cell growth and colony formation, and *MNAT1-*knockdown dramatically decreased cell motility and invasion. MNAT1 physically interacted with p53, MNAT1 also increased the interaction of MDM2 with p53. Strikingly, MNAT1 mediated p53 ubiquitin-degradation. MNAT1 shortened p53 half-life, and ectopic MNAT1 expression decreased p53 protein stability. Moreover, MNAT1 induced RAD51 and reduced p21, cleaved-caspase3, cleaved-PARP and BAX expression. MNAT1 inhibited CRC cell apoptosis. shMANT1 decreased tumor growths in nude mice following p53 increase.

The article "MNAT1 is overexpressed in colorectal cancer and mediates p53 ubiquitin-degradation to promote colorectal cancer malignance" was retracted in 2021. Reasons: duplicated images; unreliable data; lack of ethics approval or compliance; concerns about the data.

**Conclusion:**

MNAT1 binds to p53, mediates p53 ubiquitin-degradation through MDM2, increases cell growth and decreases cell apoptosis, and finally promotes CRC malignance. MNAT1 binding to p53 and mediating p53 ubiquitin-degradation axis represents a novel molecular joint in the p53 pathway.

**Electronic supplementary material:**

The online version of this article (10.1186/s13046-018-0956-3) contains supplementary material, which is available to authorized users.

## Background

Colorectal cancer (CRC) is one of the most common malignancies worldwide, with approximately 1.2 million new cases and 608,700 deaths every year [1]. Various factors are involved in CRC incidence. CRC development is characterized by an ‘adenoma– carcinoma sequence’. Overexpression of specific oncogenes or low expression of tumor suppressor genes in the epithelium results in the formation of a hyperproliferative mucosa, produces a benign adenoma, and eventually forms a carcinoma [2–4]. This process is orchestrated by different proteins, such as, Wnt, bone morphogenetic protein (BMP) and transforming growth factor (TGF)-β, along with p53 [5]. Alterations molecule pathways, such as cell cycle, cell proliferation, and apoptosis are involved in CRC onset. These alterations are responsible for colorectal epithelium carcinogenesis, which evenly confer individual susceptibility to cancers when they are germlines [6–8].

MNAT1 (menage a trois 1, MAT1) was initially identified as the third subunit besides CDK7 and Cyclin H in cyclin-dependent kinase-activating kinase (CAK) complex [9–12]. MNAT1 functions as an assembly factor and a substrate specificity-determining factor of CAK to promote the stability and activation of CAK [13–15]. Moreover, CAK, as the kinase subunit of general transcription factor IIH (TFIIH), is involved in transcription [10]. Activated CAK implicates in phosphorylating and activating CDKs to ensure cell cycle progression [16], phosphorylating retinoblastoma tumor suppressor protein (pRb) to mediate cell cycle G1 exit [17–19]. Importantly, CAK can phosphorylates a series of transcription factors, including p53, Oct-1, Oct-2, Oct-3, retinoic acid receptor alpha (RARα), and peroxisome proliferator-activated receptor gamma (PPARγ), thereby regulating gene transcription [14, 15]. MNAT1 exerts the above functions through its distinct domains interacting with downstream molecules. C-terminal domain of MNAT1 interacts with the CDK7-Cyclin H complex to stimulate CDK7 kinase activity, the coiled-coil domain of MNAT1 interacts with XPD and XPB to anchor CAK to TFIIH core, while N-terminal domain RING finger of MAT1 is involved in C-terminal domain (CTD) phosphorylation of RNA Polymerase II (PolII), which is required for gene promoter release and transcription initiation [20]. Intact MNAT1 expression is associated with cell cycle G1 exit, whereas intrinsically programmed or RA-induced MNAT1 degradation leads to cell cycle arrest, transcription inhibition and cell differentiation [18, 21–23]. In the inhibition of RA-induced granulocytic differentiation, an inhibition of MNAT1 degradation mediates p21 expression suppression [23]. Suppressed MNAT1 triggers apoptosis [17]. In contrast, MNAT1 overexpression is associated with low p21 expression [24]. Recent reports show that MNAT1 is overexpressed in breast cancer, its expression level is associated with ER expression and patient outcome [25]. In the present study, we found that MNAT1 is highly expressed in CRC tissues, its expression was associated with CRC carcinogenesis and poor patient outcomes. Further experiments showed that MNAT1 increases CRC cell growth in vitro and in vivo, its mechanism is that MNAT1 induces p53 ubiquitin-degradation.

The article "MNAT1 is overexpressed in colorectal cancer and mediates p53 ubiquitin-degradation to promote colorectal cancer malignance" was retracted in 2021. Reasons: duplicated images; unreliable data; lack of ethics approval or compliance; concerns about the data.

## Methods

### Reagents and antibodies

Chemical reagents for molecular biology were purchased from Sigma-Aldrich (St. Louis, MO). Dulbecco’s modified Eagle medium (DMEM) and other supplements were obtained from Life Technologies (Rockville, MD). Antibodies against p53, p21, PARP, cleaved-PARP, RAD51, caspase3, cleaved-caspase3, BAX, MDM2, and BCL-2 were purchased from Abnova Company (Shanghai, China). Antibodies against MNAT1, HSP70, GAPDH, HA and Flag were purchased from Santa Cruz Biotechnology, Inc. (Santa Cruz, CA) and Cell Signal Technology, Inc. (Beverly, MA).

### Tissue microarray and immunohistochemical staining

Human tissue microarrays containing 80 pairs of CRC tissues and corresponding adjacent non-tumor tissues, and 20 cases of CRC cancers at various stages were purchased from Outdo Biotech Company (Shanghai, China). One hundred patients enrolled into this study contained 57 males and 43 females. The median age of the patients was 46.5 age years (range 35–76), < 50 age year patients were 34 cases, > 50 age years patients were 66 cases. The tumor histology and stages were classified according to the WHO classification and the TNM staging system of the UICC, respectively. Patients in T1-T2 stages were 37 cases, and T3-T4 patients were 63 cases. Patients in N0 stage were 39 cases, and N1-N3 patients were 61 cases. Patients in M0 stage were 34 cases, and M1 patients were 66 cases. These tissue microarrays (HcolA180su10) were stained with MNAT1 antibody (dilution 1:5000) as described previously [26]. The stained tissue microarrays were evaluated independently by two pathologists who were blinded to the clinical features and clinical outcome. Each case was scored based on the intensity and percentage of cells. At least 10 high-power fields were chosen randomly, and > 1000 cells were counted for each section. The intensity of MNAT1 staining was scored as 0 (no signal), 1+ (weak), 2 (moderate), and 3 (marked). Percentage scores were assigned as 0, negative; 1, 1–25%; 2, 26–50%; 3, 51–75%; and 4, 76–100%. The summed (extension + intensity) was used as the total score. We grouped all samples into the high expression group (total score ≥ 2) and the low one (total score<2) according to the protein expression [27]. Immunohistochemical staining for MNAT1 was quantified using German semiquantitative scoring system as described previously [28]. Immunoreactive score (IRS) was determined using the product of the extent score and the staining intensity score.

The article "MNAT1 is overexpressed in colorectal cancer and mediates p53 ubiquitin-degradation to promote colorectal cancer malignance" was retracted in 2021. Reasons: duplicated images; unreliable data; lack of ethics approval or compliance; concerns about the data.

### Cell lines and cell culture

CRC cell lines, SW480, HT-29, SW620, DLD1, HCT116, loVo, RK0, HCT116 p53^+/+^, HCT116 p53^−/−^, and HEK293T (an embryonic kidney cell line 293 T) were obtained from American Type Culture Collection (Maryland). All the cell lines were grown in DMEM supplemented with 10% fetal bovine serum (FBS) at 37 °C and in 5% CO_2_.

### Plasmids and vectors constructing

*MNAT1* DNA fragment was generated by polymerase chain reaction (PCR) and cloned into pSIN-vector containing a FLAG, HA or V5 tag sequence. *PT53* was generated using PCR and cloned into vector containing HA or FLAG. Short hairpin RNAs (sh) target *MNAT1*, and shMDM2 targets *MDM2.* shMNAT1^#^1 and shMNAT1^#^2 were designed, and shMNAT1 and shMNAT1#2 sequences are shown in Additional file 1: Table S1. shMDM2 was designed as described previously [29]. They were synthetized by GenePharma (Shanghai, China) and cloned into pLVX, and then pLVX-shMNAT1#1 and pLVX-shMNAT1#1 were obtained. HA-tagged ubiquitin was gifted by Dr. Helen Piwnica-Worms (Washington University, St. Louis). As described previously [14, 30], the vectors containing various *PT53* and *MNAT1* domains were generated using Quick-Change Site-Directed Mutagenesis Kit (Stratagene, California). PCR primers used are listed in Additional file 2: Table S2. All the mutations were verified by performing sequencing.

### Gene transfection and stable transfect of cells

Gene transfection and stable cell line establishment were performed as described previously [31]. Briefly, 1 × 10^4^ of HCT116 and DLD1 cells were transfected with 2 μg DNA of pSIN, pSIN-MNAT1, pLVX-shMNAT#1, pLVX-shMNAT1#2 or pLVX-shscramble following the manufacture’s suggested protocol. HEK293T cells were transfected with pSIN or pSIN-MNAT1. The stably transfected cell lines, pSIN-HCT116, MNAT1-HCT116, pSIN-DLD1, MNAT1-DLD1, shscramble-HCT116, shMNAT1^#^1-HCT116, shMNAT1^#^2-HCT116, shscramble-DLD1, shMNAT1^#^1-DLD1, shMNAT1^#^2-DLD1, pSIN-HEK293T, and pSIN-MNAT1-HEK293T were obtained by selection and further confirmed by assessing MNAT1 expression.

The article "MNAT1 is overexpressed in colorectal cancer and mediates p53 ubiquitin-degradation to promote colorectal cancer malignance" was retracted in 2021. Reasons: duplicated images; unreliable data; lack of ethics approval or compliance; concerns about the data.

### Western-blotting and immunoprecipitation

Western-blotting and immunoprecipitation were performed as described previously [31]. Briefly, 1 × 10^6^ cells were lysed with lysis buffer [1 × PBS, 1% Nonidet P-40, 0.5% sodium deoxycholate, 0.1% SDS, and freshly added 100 μg/ml phenylmethanesulfonyl fluoride (PMSF), 10 μ g/ml aprotinin, and 1 mM sodium orthovanadate]. Cell lysates obtained were centrifuged, and protein concentration of the clarified lysates was measured using Easy II Protein Quantitative Kit (BCA). 40 μg of the supernatant protein was separated by 10% SDS-PAGE and transferred onto a nitrocellulose membrane. The blot was blocked with 5% non fat milk, incubated with the indicated antibody, and then incubated with an appropriate peroxidase conjugated secondary antibody. The signal was developed using 4-chloro-1-napthol/3,3-o-diaminobenzidine, and relative photographic density was quantified by a gel documentation and analysis system. GAPDH or HSP70 was used as an internal control to verify basal expression levels and equal protein loading. The ratio of the specific proteins to GAPDH orHSP70 was calculated. 100 μg of the clarified supernatants were immunoprecipitated using anti-FLAG-agarose or anti-HA-agarose antibody (Sigma Chemical Co.). MNAT1 or p53 in the immunoprecipitated complexes was respectively determined by Western-blotting with anti-MNAT1 or anti-p53 antibody.

### Apoptosis analysis

Apoptosis analysis was performed as described previously [32]. Briefly, 1 × 10^4^ cells of shscramble-HCT116, shMNAT1^#^1-HCT116, shMNAT1^#^2-HCT116, pSIN-HEK293T, and pSIN-MNAT1-HEK293T were seeded on six-well plates and cultured to reach 70% confluence, and were treated with 10 or 80 μg/ml 5-fluorouracil (5-FU). After 24 h treatment, the cells were collected by 0.02% trypsin without eathylene diamine tetra acetic acid (EDTA), and stained with annexin V-EGFP (Enhanced Green Fluorescent Protein) and propidium iodide (KeyGen Biotec) according to the manufacturer’s recommendations, and analyzed by flow cytometry.

### MTT and colony formation assays

Cell growth was determined by performing MTT [3-(4,5-dimethyl-2-thiazolyl)-2,5-diphenyl-2 -H-tetrazolium bromide] assays as described previously [33]. Briefly, pSIN-HCT116, pSIN-MNAT1-HCT116, pSIN-DLD1, pSIN-MNAT1-DLD1, shscramble-HCT116, shMNAT1^#^1-HCT116, shMNAT1^#^2-HCT116, shscramble-DLD1, shMNAT1^#^1-DLD1, and shMNAT1^#^2-DLD1 cells (1 × 10^3^) were seeded in 96-well microplates. The cells were cultured for the indicated time, followed by incubation with MTT for 4 h. Optical density (OD) was determined at 450 nm using a microplate reader. Measurements were acquired once per day for 5 d. For the colony-formation assay, the cells were plated at a density of 500 cells/well in six-well plates and were cultured for 12 d. Colonies were fixed in methanol, stained with 0.5% gentian violet, and counted [34]. Results are presented as mean ± SD of three independent experiments.

The article "MNAT1 is overexpressed in colorectal cancer and mediates p53 ubiquitin-degradation to promote colorectal cancer malignance" was retracted in 2021. Reasons: duplicated images; unreliable data; lack of ethics approval or compliance; concerns about the data.

### Real-time PCR

Real-time PCR was performed as described previously [30]. Briefly, 1 μg DNase-treated RNA was reverse transcribed using Revert AidTM First-Strand cDNA Synthesis Kit (MBI Fermentas, USA) according to the manufacturer’s instructions. Threshold cycle (Ct) value of each sample was determined using Platinum SYBR Green qPCR SuperMix-UDG with ROX (Invitrogen) in ABI 7900HT Real-Time PCR System (Applied Biosystems, Foster City, CA). Sequences of primers used are shown in Additional file 3: Table S3. Relative mRNA expression of each target gene was normalized to the expression of the housekeeping gene GAPDH. Relative mRNA level was calculated as two power values of ΔCt (Ct value of GAPDH Ct of target gene).

### Tumor growth assays in vivo

In vivo tumor growth assays were performed as described previously [35]. Briefly, female BABL/c athymic nude mice (age 4 w) were obtained from an animal center of Guangdong Province (Guangzhou, China). All animal experiments were performed according to the National Institutes of Health Animal Use Guidelines on the Use of Experimental Animals. The nude mice were subcutaneously injected 2 × 10^6^ cells shscramble-HCT116, shMNAT1^#^1-HCT116p53^+/+^ or shMNAT1^#^1-HCT116p53^−/−^, 6 mice per group. Tumor sizes of nude mice were measured every 2 or 3 d, and tumor volume was estimated. After 17 days, the mice were euthanized, and the tumors were removed and weighed.

### Cell invasion and motility assay

Cell invasion and motility were assayed according to the methods described previously with minor modifications [36]. Cell invasion and motility of shscramble-HCT116, shMNAT1^#^1-HCT116, shscramble-DLD1, and shMNAT1^#^1- DLD1 cells were detected using Boyden chamber invasion assay in vitro. Briefly, for invasion assay, matrigel (25 mg/50 ml, Collaborattiv Biomedical Products, Bedford, MA) was added into the chamber to be 8 mm pore size polycarbonate membrane filters. The cells were trypsinized to be suspension cells, and were seeded into the Boyden chamber (Neuro Probe, cabin John, MD) at the upper part at a density of 1.5 × 10^4^ cells/well in 50 μl of serum-free medium, and then incubated for 12 h at 37 °C. The bottom chamber also contained standard medium with 20% FBS. The cells invaded to the lower surface of membrane were fixed with methanol and stained with hematoxylin and eosin. Invaded cell numbers were counted under a light microscope. The motility assay was carried out as described in the invasion assay with no coating of matrigel.

The article "MNAT1 is overexpressed in colorectal cancer and mediates p53 ubiquitin-degradation to promote colorectal cancer malignance" was retracted in 2021. Reasons: duplicated images; unreliable data; lack of ethics approval or compliance; concerns about the data.

### Protein half-life detection

Protein half-life was determined as described previously [37]. Briefly, pSIN- and pSIN- MNAT1-HEK293, shscramble- and shMNAT1^#^1- LoVo cells were treated with 10 mg/mL cycloheximide (CHX), and the treated cells were collected at indicated time points after CHX treatment for 0, 20, 40, 60, 90 and 120 min. Protein of the collected cells was extracted for performing Western-blotting with anti-p53 or anti-MNAT1 antibody. GAPDH was used as an internal control to verify basal level expression and equal protein loading. The abundance ratio to HSP70 was counted, and half-life time of the proteins was calculated.

#### Ubiquitination assay

In vivo ubiquitination assay was performed as described previously [37, 38]. Briefly, HEK293T cells were stable transfected with pSIN-MNAT1, LoVo cells were stable transfected with shscramble, shMNAT1^#^1 or shMNAT1^#^2. The stable cell lines were cotransfected with plasmids expressing 3Flag-p53 and HA-ubiquitin. The cells were lysed in lysis buffer. The cell lysates were centrifuged. The supernatants were immunoprecipitated with anti-Flag agarose, and the immunocomplexes were immunoblotted using anti-HA antibody.

## Results

### MNAT1 is highly expressed in CRC cells and tissues

To clarify MNAT1 expression in CRC cells, CRC cell lines, SW480, HT-29, SW620, DLD1, RK0, LoVo, and HCT116 cells were detected MNAT1 expression using Western-blotting. Compared with HEK293T, MNAT1 protein levels were mostly elevated in SW480, HT-29, SW620, DLD1, RK0, LoVo, and HCT116 (Fig. 1a). HCT116 and DLD1 had a relatively low MNAT1 expression, and LoVo had a high expression (Fig. 1a), they were used to perform the next experiments. To clarify whether MNAT1 overexpresses in CRC tissues, a tissue microarray containing 80 pairs of CRC, adjacent non-tumor tissues, and other 20 CRC tissue samples was used to detect MNAT1 expression. The immunohistochemical results showed that MNAT1 was significantly high in CRC tissues when compared with the matched adjacent normal tissues (Fig. 1b, c. *p* = 0.042). The positive rates of MNAT1 expression were compared in normal colorectal, primary CRC, and metastatic CRC tissues. The positive rates of MNAT1 were 11.3% in normal tissues, 55.9% in primary CRC and 56.1% in metastatic CRC tissues, respectively (Table 1). MNAT1 was significantly upregulated in primary CRC (Table 1. *p* = 0.031) and metastatic CRC tissues (Table 1. *p* = 0.033), whereas no difference of MICAL2 between primary CRC and metastatic CRC tissues. In addition, MNAT1 level may be used for the CRC diagnosis, and the area under the curve (AUC) was calculated. Cut off of MNAT1 was 4.6 (Fig. 1d. AUC = 0.933, *p* = 0.013). Sensitivity was 87.6%, and specificity was 67.7%. The association of MNAT1 expression with CRC stages was analyzed. MNAT1 expression was not correlated with T stage (original tumor size and nearby tissue invasion) (Table 2. *p* = 0.882), N stage (lymph node metastasis) (Table 2. *p* = 0.891), nor M stage (distant metastasis) (Table 2. *p* = 0.897). The patients with high MNAT1 displayed shorter overall survival than low MNAT1 expression (Fig. 1E, *p* = 0.011). These data strongly suggest that high MNAT1 has oncogenic potency and is associated with CRC poor outcomes.

The article "MNAT1 is overexpressed in colorectal cancer and mediates p53 ubiquitin-degradation to promote colorectal cancer malignance" was retracted in 2021. Reasons: duplicated images; unreliable data; lack of ethics approval or compliance; concerns about the data.

**Fig. 1:** MNAT1 expressions in CRC and its association with CRC patient outcomes. A, MNAT1 expressions were detected in SW480, HT-29, SW620, DLD1, RK0, LoVo, HCT116, and HEK329T using Western-blotting. B, MNAT1 expressions in CRC and non-tumor tissues microarray were detected using immunohistochemstry (IHC). a, negative, scored as 0; b, weakly positive, scored as 1; c, moderately positive, scored as 2; d, positive, scored as 3; e, positive, scored as 4; Scale Bar, 100 μm. C, MNAT1 expression levels in CRC tissue samples were quantified using a German semiquantitative scoring system. Relative expressions in CRC tissues and non-tumor tissues were statistically analyzed using Mann-Whitney *U* test. The dots represent scores. D, The cut-off value of MNAT1 immunoreactive score is 4.6 according to the ROC curve, and the AUC is 0.933. ROC, receiver operating characteristic; AUC, area under the curve. E, The overall survival of CRC patients with high (49) or low (51) MNAT1 expression. *, *p* < 0.05

**Table 1:** MNAT1 expressions in normal colorectal, primary CRC, and metastatic CRC tissues

		MNAT1			
	*n*	–	+	%	*P*
NC	80	71	9	11.3	
CRC	59	22	33	55.9	0.031^a^
MCRC	41	17	23	56.1	0.033^b^

*NC* normal colorectal tissue, *CRC* primary CRC, *MCRC* metastatic CRC tissues

^a^CRC versus NC; ^b^MCRC versus NC

**Table 2:** MNAT1 expressions in CRC samples at various clinical stages

Characteristic	Cases	MNAT1 expression		*p*
		Low(%)	High(%)	
All patients				
Gender				
Male	57	35(61.4)	22(38.6)	0.817
Female	43	29(67.4)	14(32.6)	
Age (yrs)				
< 50	34	16(47.1)	18(52.9)	0.770
≥ 50	66	35(53.0)	31(47.0)	
T stage				
T1-T2	37	19(51.3)	18(48.7)	0.882
T3-T4	63	34(53.9)	29(46.1)	
N stage				
N0	39	17(43.6)	22(56.4)	0.891
N1-N3	61	29(47.5)	32(52.5)	
M stage				
M0	34	18(52.9)	16(47.1)	0.897
M1	66	35(53.0)	31(47.0)	

The article "MNAT1 is overexpressed in colorectal cancer and mediates p53 ubiquitin-degradation to promote colorectal cancer malignance" was retracted in 2021. Reasons: duplicated images; unreliable data; lack of ethics approval or compliance; concerns about the data.

### Oncogenic properties of MNAT1 in CRC cells

HCT116 and DLD1 cells with low MNAT1 expressions were used to investigate MNAT1 function in CRC cell growth. We constructed MNAT1 expression vector, pSIN-MNAT1. HCT116 and DLD1 cells were transfected with pSIN-MNAT1. MNAT1 was detected in the transfected cells using Western-blotting, and the results displayed that MNAT1 was overexpressed in the transfected cells (Fig. 2A). Viability of the transfected cells was determined by performing MTT assay. MTT data showed that the growth kinetics of HCT116 (Fig. 2B-a. *p* < 0.05) and DLD1 cells (Fig. 2B-b. *p* < 0.05) increased when being transfected with MNAT1. Further, cell colony formation of the transfected cells was detected. MNAT1 dramatically increased colony formation of HCT116 (Fig. 2C-a, b, c. *p* < 0.05) and DLD1 cells (Fig. 2C-d, e, f. *p* < 0.05). Next, shMNAT1^#^1 and shMNAT1^#^2 were designed to target MNAT1, and pLVX-shMNAT1^#^1 and pLVX-shMNAT1^#^2 were constructed. HCT116 and DLD1 were infected with pLVX-shMNAT1^#^1 and pLVX-shMNAT1^#^2. Western-blotting and real-time PCR were performed to evaluate the efficiency of shMNAT1^#^1, 2. The results showed that the shMNAT1^#^1, 2 effectively blocked MNAT1 protein (Fig. 2D-a) and mRNA expression (Fig. 2D-b, c). After MNAT1 was knockdown, HCT116 (Fig. 2E-a, *p* < 0.05) and DLD1 (Fig. 2E-b, *p* < 0.05) growths were decreased when compared with the scramble control. Simultaneously, motility and invasion of the transfected cells were also observed, 10 fields were randomly selected and counted the invaded cells per cell well. The results showed that the motility and invasion of MNAT1-knockdown cells were dramatically decreased when compared with the scramble group (Fig. 2F-a, b, c; Fig.2G-a, b, c. *p* < 0.05).

**Fig. 2:** MNAT1 increases CRC cell growth and *MNAT1*-knockdown decreases cell growth. HCT116 and DLD1 cells were transfected with pSIN-MNAT1 respectively. A, MNAT1 expressions in the transfected cells were detected using Western-blotting. B, Viability of MNAT1 transfected-HCT116 (a) and DLD1 (b) cells was measured using MTT. C, Colony formation of the transfected- HCT116 and DLD1 cells was detected using colony formation assay. a, HCT116 with pSIN; b, HCT116 with pSIN-MNAT1; c, Cell colony numbers of the transfected HCT116; d, DLD1 with pSIN; e, DLD1 with pSIN-MNAT1; f, Cell colony numbers of the transfected DLD1. D, HCT116 and DLD1 cells were transfected with pLVX-shMNAT1^#^1or pLVX-shMNAT1^#^2, respectively. MNAT1 protein (a) and mRNA (b, c) in the transfected cells were detected using Western-blotting or Real-time PCR, respectively. E, Viability of shMNAT1 transfected-HCT116 (a) and DLD1 (b) cells was measured using MTT. F, Motility and invasion of HCT116 cells with shMNAT1s were detected with Boyden chamber invasion assay (a), the motility (b) and invasion (c) cells were counted. G, Motility and invasion of DLD1 cells with shMNAT1s were detected (a), the motility (b) and invasion (c) cells were counted. All experiments were repeated three times. Data are presented as means ±S.D. of three independent experiments and were statistically analyzed using Student’s t test. Scale bar, 100 μm. *, *p* < 0.05

The article "MNAT1 is overexpressed in colorectal cancer and mediates p53 ubiquitin-degradation to promote colorectal cancer malignance" was retracted in 2021. Reasons: duplicated images; unreliable data; lack of ethics approval or compliance; concerns about the data.

### MNAT1 down-regulates expressions of p53

The above results suggested that MNAT1 is associated with CRC cell growth. We next investigated mechanisms underlying MNAT1-regulated cell growth, and focused on MNAT1 regulating p53 and its molecular mechanism. CRC cells were transfected with MNAT1 expression vectors, p53 and *PT*53 mRNA expressions were detected. The results showed that p53 expressions significantly decreased after being transfected with MNAT1 (Fig. 3A-a, b), but p53 mRNA expression did not change (Fig. 3B). To observe the dose effect of MNAT1 on p53 expression, HEK293T cells were exogenously transfected HA-p53 and various dose Flag-MNAT1, and then p53 was detected. p53 expression decreased along with MNAT1-dose increase, displaying a dose-dependent manner (Fig.3C-a, b). To further observe the effect of MNAT1 silencing on p53 expression, LoVo cells were transfected with shMNAT1#1 and #2, and p53 expression was detected. The results showed that p53 expression was increased when MNAT1 was silenced (Fig. 3D). Doxorubicin (DOX), an anticancer regent, has been proved to increase p53 expression [39]. Dox was used to treat HCT116 cells at various concentrations, and p53 and MNAT1 expressions were analyzed. MNAT1 gradually decreased along with DOX concentration increase, while p53 gradually increased, displaying significantly concentration-dependent (Fig. 3E). In the next, HCT116 cells were transfected with pSIN-MNAT1, and then the transfected cells were treated with MG132, a specific proteasome inhibitor to inhibit MNAT1 expression, and p53 expression was observed. MG132 substantially rescued the raise of p53 protein level caused by pSIN-MNAT1 (Fig. 3F), further this results were confirmed with DOX reducing MANT1 expression (Fig. 3G). These suggest that MNAT1 decreases p53 expression by the proteasome.

**Fig. 3:** MNAT1 decreases p53 expression. A, HCT116 cells were transfected with Flag-MNAT1 (a), and DLD1 cells were transfected with pSIN-MNAT1 (b), p53 expressions the tranfected cells were detected using Western-blotting. B, *PT53* mRNA expressions in the transfected cells were detected using Real-time PCR. C, HEK293T cells were cotransfected with HA-p53 and Flag-MNAT1 at various concentrations, Flag and HA expressions were detected (a). Abundances of Flag and HA were analyzed (b). D, LoVo cells were transfected with shsramble, shMNAT1#1 and #2, and then p53 and MNAT1 expressions in the transfected cells were detected using Western-blotting. E. LoVo cells were treated with COX at the indicated concentrations, and then MNAT1 and p53 expressions were detected. F, HEK293T cells were transfected with pSIN-MNAT1 or blank vector, and then treated with DOX. MNAT1 and p53 expressions were detected using Western-blotting. G, HEK293T cells transfected with pSIN-MNAT1 were treated with DOX and/or MG132, and then MNAT1 and p53 were detected. DOX, Doxorubicin; *, *p* < 0.05

The article "MNAT1 is overexpressed in colorectal cancer and mediates p53 ubiquitin-degradation to promote colorectal cancer malignance" was retracted in 2021. Reasons: duplicated images; unreliable data; lack of ethics approval or compliance; concerns about the data.

### MNAT1 interacts with p53

In this step, we first performed endogenous immunoprecipitation assay to examine whether MNAT1 directly interacted with p53. LoVo cells with high expression MNAT1 were used to immunoprecipitate p53 and MNAT1, and then p53 and MNAT1 were detected in the immunocomplexes using Western-blotting. The results showed that p53 was detectable in MNAT1-immunoprecipitated complexes, and MNAT1 was also detectable in p53 immunocomplexes (Fig. 4A). To further confirm the interaction of MNAT1 with p53, HEK293T cells were contransfected with HA-p53 and Flag-MNAT1, and then their interaction was determined using immunoprecipitation. Immunoprecipitation results showed that MNAT1 bound to p53 (Fig. 4B). These findings indicated that MNAT1 interacts with p53. Next, we determined the domains of p53 involved in this interaction using p53- and MNAT1-expressing plasmids. The plasmids expressing various p53 domains were constructed (Fig. 4C-a). HEK293T cells were transfected with the indicated plasmids, and the immunoprecipitation was performed to identify the interacting domains of p53. The results showed that the domains containing residue 1–300 displayed a binding band with MNAT1, while the deletion of residues 100–300 had no binding signal (Fig. 4C-b). This indicated that the domain of p53 residues 100–300 was necessary and sufficient for interaction with MNAT1. Simultaneously, to determine the domains of MNAT1 participated in the binding of MNAT1 to p53, the plasmids containing various MNAT1 domains were constructed (Fig. 4D-a) and the plasmids were transfected into HEK293T cells, the immunoprecipitation was performed to identify the interacting domains of MNAT1. The results showed that only full-long MNAT1 interacted with p53, and MNAT1 mutants containing domain deletion could not interact with p53 (Fig. 4D-b).

The article "MNAT1 is overexpressed in colorectal cancer and mediates p53 ubiquitin-degradation to promote colorectal cancer malignance" was retracted in 2021. Reasons: duplicated images; unreliable data; lack of ethics approval or compliance; concerns about the data.

**Fig. 4:** MNAT1 interacts with p53. A, the lysates of LoVo cells were immunoprecipitated using anti-IgG, anti-MNAT1 or anti-p53 antibodies, and immunoprecipitation products were analyzed by Western-blotting with the indicated antibody. B, HEK293T cells were cotransfected with Flag-MNAT1 and HA-p53. Flag or HA was immunoprecipitated in the transfected cells, and the immunocomplexes were detected using Western-blotting with HA- or Flag-antibody. C, The various construct plasmids of *TP53* were constructed using PCR (a)*.* HEK293T cells were cotransfected with Flag-MNAT1 and the indicated plasmids of *TP53*. Immunoprecipitation was performed using anti-HA antibody, and the immunoprecipitated products were detected using Western-blotting with anti-Flag antibody. D, The plasmids containing various *MNAT1* gene segments were constructed (a). HEK293T cells were cotransfected with HA-*TP53* and the indicated plasmids of Flag-MNAT1. Immunoprecipitation was performed using anti-Flag antibody, and the immunoprecipitated products were detected using Western-blotting with anti-HA antibody. FL, full length p53; IP, immunoprecipitation; WCL, whole cell lysate

### MNAT1 promotes ubiquitin-degradation of p53

The above results suggest that MNAT1 decreases p53 protein level, while p53 mRNA level did not change, indicating that MNAT1 may regulate p53 at post-transcriptional level. We speculated that MNAT1 affects p53 proteolysis. To confirm this, HEK293T cells were co-transfected with v5-MNAT1 and Flag-p53, and then p53-ubiquitin was detected. The results showed that Flag-p53 poly-ubiquitin was stronger in the MNAT1 transfect than the blank control (Fig. 5a). Further, we used shMNAT1 to knockdown MNAT1 expression, and observed whether the reduced-MNAT1 decreases p53 ubiquitination. The results showed that Flag-p53 ubiquitination was dramatically decreased when being transfected shMNAT1 (Fig. 5b). Additionally, we investigated whether MNAT1 could exactly mediate endogenous p53 ubiquitination. pSIN-MNAT1 was transfected into HCT116, and p53 ubiquitination was observed. The endogenous p53 ubiquitination significantly increased when transfected with pSIN-MNAT1 (Fig. 5c). We also observed the effect of MANT1*-*knockdown on endogenous p53 ubiquitination. p53 ubiquitin-degradation dramatically decreased (Fig. 5d), and the cotransfection with shMNAT1^#^1 and shMNAT1^#^2 had less p53 ubiquitin-degradation than the single one (Fig. 5e). The rescue experiments of MNAT1-mediated p53 ubiquitin-degradation were performed. MANT1-HEK293 cell was treated with MG132, and then p53 ubiquitination was detected. The results showed that p53 ubiquitin-degradation significantly increased in the MNAT1- transfected cell, this p53 ubiquitin-degradation was decreased by MG132 treatment (Fig. 5e). Collectively, these results indicate that MNAT1 increases p53 ubiquitination, thus promoting its proteasomal degradation.

The article "MNAT1 is overexpressed in colorectal cancer and mediates p53 ubiquitin-degradation to promote colorectal cancer malignance" was retracted in 2021. Reasons: duplicated images; unreliable data; lack of ethics approval or compliance; concerns about the data.

**Fig. 5:** MNAT1 promotes p53 ubiquitin-mediated degradation. A, HEK293T cells were cotransfected with HA-Ub, Flag-p53, and v5-MNAT1. Flag was immunoprecipitated in the transfected cells, and p53 was detected using Western-blotting (a), and p53 life-time was calculated (b). B, LoVo cells were cotransfected with HA-Ub, Flag-p53 and pLVX-shMNAT1^#^1 or pLVX-shMNAT1^#^2, respectively. The transfected cells were immunoprecipitated with Flag antibody, and p53 in the immunocomplexes were detected. C, HCT116 cells were cotransfected with pLVX-shMNAT1^#^1 or pLVX-shMNAT1^#^2, respectively. The transfected cells were immunoprecipitated with p53 antibody, and then ubiquitin in the immunocomplexes was detected. D, HEK293 cells were transfected with pSIN-MNAT1, and p53 in the transfected cells was immunoprecipitated. Ubiquitin in the immunocomplexes was detected. E, HCT116 cells were cotransfected with pLVX-shMNAT1^#^1 and ^#^2. p53 in the transfeccted cells was immunoprecipitated, and its ubiquitination was detected. IP, immunoprecipitation; Ub, ubiquitin; WCL, whole cell lysate

### MNAT1 shortens half-time p53

The above findings showed that MNAT1 promotes p53 ubiquitin-degradation. Moreover ubiquitin-proteasome is a highly effective protein-degradation pathway in eukaryotic cells [40–42]. Next step, we detected the half-life time of p53 when MNAT1 knockin and MNAT1 knockout. HEK293 cells were transfected with pSIN-MNAT1, and treated with CHX. The half-life time of endogenous p53 protein was measured in the treated cells. The half-life time of endogenous p53 was shorter in the transfect with pSIN-MNAT1 than in the control cells (Fig. 6A-a, b). Simultaneously, LoVo cells were knockdown MNAT1 with shMANT1^#^1, and p53 half-life was analyzed. The data showed that p53 half-life time was longer in the cells with shMNAT1 transfection than the control (Fig. 6B-a, b). E3 ubiquitin ligase murine double minute (MDM2) is the most critical negative regulator for p53 protein stability. MDM2 binds to p53 and ubiquitinates it for proteasomal degradation [43–45]. Therefore, we tested the effect of MNAT1 on the interaction of MDM2 with p53. MDM2 binding to p53 was dramatically increased in the cells with MNAT1 transfection, while MDM2 interacted with p53 was significantly decreased when MNAT1 knockdown (Fig. 6C-a, b. *p* < 0.05). To further confirm whether MNAT1-mediated p53 decrease is through MDM2, stable cell line, MANT1-HEK293 cells were knockdown MDM2 with shMDM2 to observe p53 expression. The results showed that MNAT1 significantly decreased p53 expression, but p53 decrease was not significant when MDM2 knockdown (Fig. 6D). These data suggested MNAT1 mediates p53 ubiquitin through increasing interaction of MDM2 with p53.

The article "MNAT1 is overexpressed in colorectal cancer and mediates p53 ubiquitin-degradation to promote colorectal cancer malignance" was retracted in 2021. Reasons: duplicated images; unreliable data; lack of ethics approval or compliance; concerns about the data.

**Fig. 6:** MNAT1 shortens half-life time of p53. A, HEK293 cells were transfected with pSIN or pSIN-MNAT1, and then treated with 20 mg/ml CHX for the indicated time points. pSIN served as a control. MANT1 and p53 expressions were detected using Western-blotting (a). Quantitative analysis was conducted on p53 level in Western-blotting, the half-life time of p53 was calculated (b). B, LoVo cells were transfected with pLVX-shMNAT1^#^1, p53 and MNAT1 expressions in the transfected cells were detected (a). Quantitative analysis was conducted on p53 level, and the half-life time was also calculated (b). C, HEK293 cells were transfected with pSIN-MNAT1, and LoVo cells were transfected with pLVX-shMNAT1^#^1 or pLVX-shMNAT1^#^2. p53 was immunoprecipitated, and MDM2 was detected in the immunocomplexes and WCL using Western-blotting (a). Quantitative analysis was conducted on p53 and MNAT1 expressions (b). D, MANT1-HEK293 cells were transfected with shMDM2, and p53, MDM2, MNAT1 expressions were detected in the transfected cells. CHX, cycloheximide; IP, immunoprecipitation; MGM2, murine double minute 2. WCL, whole cell lysate. *, *p* < 0.05

### MNAT1 regulates p53 downstream genes

The above findings showed that MNAT1 decreases p53 through ubiquitin-degradation. In the next step, we investigated whether MNAT1-decreased p53 affects p53 downstream genes. HEK293T cells were transfected with pSIN-MNAT1, and then p53, p21, caspase, PARP, RAD51, BAX, and Bcl2 were tested. p53, p21, cleaved- caspase 3, cleaved-PARP and BAX were decreased in the transfected cells, and RAD51 was increased (Fig. 7A). To further probe whether MNAT1 regulating p21, PAPR, BAX, and RAD51 is through p53, HCT116 p53^+/+^ and HCT116 p53^−/−^ cells were used to determine whether *p53* gene is essential. The results showed that MNAT1-knockdown increased p53, p21, and BAX expressions, and decreased PARK and RAD51 expression in HCT116 p53^+/+^, did not in HCT116 p53^−/−^ cells (Fig. 7B). DOX is an anticancer regent, it has proved to inhibit synthesis of RNA and DNA [46]. The previous data showed that DOX inhibits MNAT1 expression. To further clarify whether DOX decreased-MNAT1 also regulates p53 downstream molecule, HCT116 cells were transfected with shMNAT1 or pSIN-MNAT1, and then treated with DOX. The results showed that the cleaved PARP was not increased when transfected with MNAT1, but cleaved PARP was increased when being transfected with shMANT1 (Fig. 7C). Whether 5-FU-reduced MNAT1 regulates p53 downstream molecules was investigated. Fas, a p53 target gene, was decreased in the transfect with MANT1, but did not change in the transfect with shMNAT1 (Fig. 7D). Simultaneously, apoptosis in MNAT1-knockdown cells was also detected, there was no difference (data not shown). So, 5-FU was used to treat MNAT1-knockdown cells, and cell apoptosis was detected using flow cytometry. The results showed that shMNAT1^#^1 and shMNAT1^#^2 significantly enhanced 5-FU-induced apoptosis (Fig. 7E-b, c, f. *p* < 0.05), and pSIN-MNAT1 reduced 5-FU-induced apoptosis (Fig. 7E-e, f. *p* < 0.05). Collectively, MNAT1 decreases p53 expression, and regulates p53 downstream molecules, reduced cell apoptosis.

The article "MNAT1 is overexpressed in colorectal cancer and mediates p53 ubiquitin-degradation to promote colorectal cancer malignance" was retracted in 2021. Reasons: duplicated images; unreliable data; lack of ethics approval or compliance; concerns about the data.

**Fig. 7:** MNAT1 regulates p53 down-stream molecules. A, HEK293T cells were transfected with pSIN or pSIN-MANT1, and then MNAT1, p53, p21, cleaved caspase3, caspase3, cleaved PARP, PARP, BAX, RAD51, and Bcl2 were detected with Western-blotting. pSIN served as a control. B, HCT116 p53^+/+^ and HCT116 p53^−/−^ cells were transfected with pLVX-shscramble, pLVX-shMNAT1^#^1 or pLVX-shMNAT1^#^2, respectively. pLVX-shscramble served as a control. MANT1, p53, p21, BAX, PARP, and RAD51 were detected. C, LoVo cells were transfected with pLVX-shMNAT1^#^1, and HEK293T cells were transfected with pSIN-MANT1. And then the transfected cells were treated with DOX. The treated cells were evaluated MNAT1, PARP, p53 expression. GAPDH served as a loading control. D, LoVo cells were infected with pLVX-shMNAT1^#^1 or pLVX-shMNAT1^#^2, and HEK293T cells were transfected with pSIN-MANT1, and then treated with 5-Fu. The treated cells were evaluated MNAT1, p53, and Fas expression. E, The apoptosis of the treated cells was analyzed using flow cytometry, and apoptosis rates were conducted. a, shscramble plus 5-FU; b, shMNAT1^#^1 plus 5-FU; c, shMNAT1^#^2 plus 5-FU; d, blank vector plus 5-FU; e, pSIN-MNAT1 plus 5-FU; f, apoptosis rates of the above treated cell. DOX, Doxorubicin; 5-Fu, 5-fluorouracil; *, *p* < 0.05

### MNAT1 promotes CRC growth in vivo

The above-mentioned results showed that MNAT1 increased CRC cell growth and colony formation, and also found MNAT1-mediated p53 ubiquitin-degradation, and regulated p53 downstream molecules. In the next step, we further confirmed whether MNAT1 exerts oncogenic effect in vivo. Shscramble-HCT116, shMNAT1^#^1-HCT116 cells were subcutaneously injected into the dorsal flanks of mice. The tumors of mice were measured per 2 d. After 17 days, the mice were euthanized, and tumor weights were measured. Data showed that the tumors of mice injected with shMNAT1^#^1-HCT116 were smaller than that of the shscramble mice (Fig. 8A, B. *p* < 0.05). MNAT1 and p53 expression was detected in these tumor tissues using immunohistochemistry, and positive cells were counted in 10 fields of the IHC stained section under microscopy. Immunohistochemical results showed that MNAT1 expression was low, and p53 was high in the tumor tissues of shMNAT1^#^1-HCT116 when compared with the shscramble group (Fig. 8C-a,b. *p* < 0.05). These results indicated that MNAT1 promoted CRC growth through down-regulating p53 in vivo*.* Summarily, MNAT1 binds to p53, and mediates p53 ubiquitin-degradation through MDM2, decreased p53 functions, and finally promotes CRC growth (Fig. 8D).

The article "MNAT1 is overexpressed in colorectal cancer and mediates p53 ubiquitin-degradation to promote colorectal cancer malignance" was retracted in 2021. Reasons: duplicated images; unreliable data; lack of ethics approval or compliance; concerns about the data.

**Fig. 8:** MNAT1 exerts tumor-promoting effects through p53 in vivo. A, shscramble-HCT116 and shMNAT1^#^1-HCT116 cells were subcutaneously injected into the dorsal flanks of mice, and shscramble-HCT116 served as a control. After 17 days, the mice were euthanized. Representative images are shown (a). After euthanization, the tumors of mice were removed. The removed tumors were weighed (b). B, The tumor growth of shscramble-HCT116 and shMNAT1^#^1-HCT116 cells in vivo was calculated by tumor volume. C, MNAT1 and p53 expressions in the implanted tumors were detected using immunohistochemistry (IHC) (a), positive cells were counted in 10 fields of the IHC stained section under microscope (b). *, *p* < 0.05. D, Schematic illustration of MNAT-promoted CRC tumorigenesis. MNAT1 binds to p53, and mediates p53ubiquitin-degaradation, and increases cell growth and decreases cell apoptosis, finally promotes CRC malignance

## Discussion

The adenoma–carcinoma multistage theory has been documented for CRC carcinogenesis. In this carcinogenesis process, mutation activating multiple oncogenes and inactivating tumor-suppressor genes accumulate in normal colonic epithelial cells and cause adenomas [4]. Our results suggest that MNAT1 is a novel gene in CRC pathogenesis. This is based upon the following three results. (1) MNAT1 was highly expressed in CRC cells, and its expression was associated with advanced CRC development and low 5-year survival rate. (2) *MNAT1* increased CRC cell malignant activity. (3) In vivo, *MNAT1-*knockdown decreases tumor growth. These results suggested that MNAT1 promotes CRC development. Determination of the underlying mechanism indicated that MNAT1 promotes CRC development through downregulating p53.

Tumor suppressor p53, encoded by *TP53* gene, is a central player in cellular DNA damage responses and is mutated in 50 to 55% of human cancers, whose primary function is to promote cell-cycle arrest and induce apoptosis when necessary [47]. p53, which is known as the guardian of the genome [48], plays a critical role in inducing apoptosis and preventing oncogenesis [49]. p53 is frequently dysregulated in CRC tissues. Moreover, p53 is associated with CRC pathogenesis and advanced TNM stage, lymph nodes metastasis, and low 5-year survival rate [50, 51]. Of the well-known functions of p53, the mostly highlighted ones are the regulation of cell cycle checkpoints and inducing apoptosis under cellular stress [52]. Loss of p53 often induces oncogenesis [53–55], and promotes tumor initiation and progression [56–58]. In the present study, we found that MNAT1 shortened p53 half-lift, suggesting that MNAT1 may promote CRC carcinogenesis through decreasing p53 function. Determination of the underlying mechanism indicated that (1) MNAT1 decreases apoptosis through reducing p53 and that (2) MNAT1 regulated p53 downstream molecules, including p21, PARK, RAD51, and FAS. p21 is critical for p53-mediated G1/S boundary cell cycle arrest [59]. p53 mediates cell apoptosis by activating mitochondrial and death receptor-induced apoptotic pathways. The mitochondrial pathway is mainly regulated by binding to Bcl-2, and releasing the cell death factors, BAX and BAK, and activate apoptosis [60, 61]. In our study, MNAT1 not only decreased BAX, but also mediated FAS increase. FAS is a component transcriptionally regulated by p53 in the extrinsic apoptotic pathway FAS [62, 63]. MANT1-mediated apoptosis inhibition may be through the extrinsic apoptotic pathway. MNAT1-mediated p21 decrease implies that MANT1 may arrest cell cycle through p21 to participate in CRC development. These remain to be further investigated.

The article "MNAT1 is overexpressed in colorectal cancer and mediates p53 ubiquitin-degradation to promote colorectal cancer malignance" was retracted in 2021. Reasons: duplicated images; unreliable data; lack of ethics approval or compliance; concerns about the data.

Interestingly, MNAT1 interacted with p53 and promoted p53 ubiquitination and degradation. MNAT1-mediated p53 degradation may be critical for CRC initiation and progression. p53 activity can be regulated through ubiquitination, oxidation, phosphorylation, acetylation and methylation [64–66]. The key to the regulation of p53 activity is the regulation of its stability, which is mainly orchestrated through a network of ubiquitination reactions [64, 65] . Among numerous proteins involved in p53 regulation, MDM2 is the major negative regulator of p53 level and activity [43, 67] . MDM2 physically interacts with p53 and represses p53-mediated transcriptional activation [44, 45] and induce p53 ubiquitination. The E3 ubiquitin ligase MDM2 is the most important regulator ubiquitin-mediated degradation of p53 [67]. MDM2 binds to p53 and ubiquitinates it proteasomal degradation [43–45]. In the present study, *MNAT1* knock-in increased MDM2 interaction with p53, and this interaction was decreased when *MNAT1* knockdown. *MDM2*-knockdown decreased MNAT1-reduced p53. These data suggest that MNAT1-mediated p53 ubiquitin-degradation is through increasing the interaction of MDM2 with p53. MDM2 may be a critical factor in MNAT1 mediated-p53 ubiquitination.

The article "MNAT1 is overexpressed in colorectal cancer and mediates p53 ubiquitin-degradation to promote colorectal cancer malignance" was retracted in 2021. Reasons: duplicated images; unreliable data; lack of ethics approval or compliance; concerns about the data.

## Conclusion

MNAT1 binds to p53, promotes p53 ubiquitin-degradation, and decreases its function. MNAT1-reduced p53 decreases CRC cell apoptosis and increases CRC cell growth both in vitro and in vivo, thus promoting CRC malignance (Fig. 8D). MNAT1 binding to p53 and mediating p53 ubiquitin-degradation axis represents a novel molecular joint in the p53 pathway.

## Additional files

Additional file 1: **Table S1.** MNAT1 shRNA sequence. (DOCX 15 kb)

Additional file 2: **Table S2.** PCR primers of plasmids construct. (DOCX 16 kb)

Additional file 3: **Table S3.** Primers of Real-time PCR. (DOCX 15 kb)

## Abbreviations

5-FU: 5-fluorouracil
AUC: Area under the curve
BMP: Bone morphogenetic protein
CAK: Kinase-activating kinase
CHX: Cycloheximide
CRC: Colorectal cancer
DOX: Doxorubicin
FBS: Fetal bovine serum
IRS: Immunoreactive score
MDM2: Murine double minute
MNAT1: Menage a trois 1
MTT: 3-(4,5-dimethyl-2-thiazolyl)-2,5-diphenyl-2-H-tetrazolium bromide
OD: Optical density
sh: Short hairpin RNAs
